# A Novel *N*-Gram-Based Image Classification Model and Its Applications in Diagnosing Thyroid Nodule and Retinal OCT Images

**DOI:** 10.1155/2022/3151554

**Published:** 2022-05-02

**Authors:** Guanfang Wang, Xianshan Chen, Geng Tian, Jiasheng Yang

**Affiliations:** ^1^Genies Beijing Co., Ltd., Beijing 100102, China; ^2^Department of Thoracic Surgery, Hainan General Hospital, Haikou, Hainan 570311, China; ^3^School of Electrical and Information Engineering, Anhui University of Technology, Maanshan, Anhui 243002, China

## Abstract

Imbalanced classes and dimensional disasters are critical challenges in medical image classification. As a classical machine learning model, the *n*-gram model has shown excellent performance in addressing this issue in text classification. In this study, we proposed an algorithm to classify medical images by extracting their *n*-gram semantic features. This algorithm first converts an image classification problem to a text classification problem by building an *n*-gram corpus for an image. After that, the algorithm was based on the *n*-gram model to classify images. The algorithm was evaluated by two independent public datasets. The first experiment is to diagnose benign and malignant thyroid nodules. The best area under the curve (AUC) is 0.989. The second experiment is to diagnose the type of fundus lesion. The best result is that it correctly identified 86.667% of patients with dry age-related macular degeneration (AMD), 93.333% of patients with diabetic macular edema (DME), and 93.333% of normal individuals.

## 1. Introduction

Medical imaging is essential in diagnosis. However, the huge amount of image data generated in exponential manner has made the image-processing task time-consuming [1]. Furthermore, factors such as irregularity, inexperience, or fatigue may lead to misdiagnosis [2].

With the rapid development of medical image acquisition and storage technology, computer-aided diagnosis (CAD) [3] systems have become an attractive option. For example, a CAD system developed by Raghavendra et al. [4] uses an optimized multilevel elongated binary model to characterize thyroid nodules. Yu et al. [5] proposed a weakly supervised segmentation neural network approach to alleviate the differences in nodule size in thyroid ultrasound images which may cause under- and/or over-segmentation problems. Koundal et al. [6] proposed an automated Intuitionistic Fuzzy Active Contour Method (IFACM) that integrates intuitionistic fuzzy clustering with the active contour for the segmentation of thyroid nodules' ultrasound images. Abdolali et al. [7] presented a novel deep neural network architecture that can detect various types of thyroid nodules. Pekala et al. [8] described a new method combining fully convolutional networks (FCN) with Gaussian processes for post processing which could be used for the automated fine-grained segmentation of spectral domain optical coherence tomography (OCT) images of the retina. Kauer-Bonin et al. [9] proposed a real-time feedback system for automatic quality assessment of retinal OCT images.

One of the most important goals of CAD is to classify medical images into different categories to help doctors in disease diagnosis or further research. It is general practice to extract features from a preprocessed image before passing them to a classifier for classification. Feature extraction and selection are key players in classifier performance. The widely used medical image features are mostly based on the underlying information of the image, such as color, texture, and shape [10]. These are content-based image classification technologies. However, the computer struggles to understand the meaning of the image from the underlying information, resulting in a “semantic gap” [11] between the “semantic similarity” of human understanding and the “visual similarity” of computer understanding.

Semantic-based classification methods, mainly deep learning-based convolutional neural network (CNN) models [12], part-based models [13], and bag-of-words (BOW) models [14], have received eager attention and application in recent years.

Among them, the CNN model avoids the feature extraction and data reconstruction process, but the model has some drawbacks in clinical applications, such as reliance on high-quality big data [15–17], weak generalization ability [18], poor interpretability [19], and high operational costs [20]. Part-based models can accurately describe the relationships between local features, but training the models is complex [21]. In 2003, Sivic and Zisserman [22] proposed the visual bag-of-words model, which introduced the bag-of-words model into the field of computer vision with great success. However, this model treated local features as independent individuals without accounting for the connection between features [23].

In general, features are classified as suitable, unnecessary, or repeated [24]. For the extracted image features, it may still have a large dimensionality and may contain certain irrelevant or redundant features. Therefore, in recent years, researchers have proposed and developed many methods and techniques to reduce the high dimensionality of data and improve model accuracy. Alharan et al. [25] proposed to evaluate the extracted features by five techniques (information gain, gain ratio, oneR, ReliefF, and symmetric). Then, based on the assessment results, feature selection was accomplished by utilizing the *K*-mean clustering algorithm. Li et al. [26] developed a radiological model based on multivariate logistic regression with the optimal 12 radiomic features after feature dimensionality reduction. The model performed well for the classification accuracy of the PTC and NG thyroid nodules in the training group and validation group. Lai and Deng [27] developed a deep learning model called Coding Network with Multilayer Perceptron (CNMP), which combines high-level features extracted from deep convolutional neural networks with some selected traditional features. In order to decipher the intrinsic structure of the benign and malignant thyroid nodule, Raghavendra et al. [28] used spatial gray level dependence features and fractal textures while Yu et al. [29] extracted 2 morphological features and 65 textural features of the region of interest to describe the thyroid nodules. Ardakani et al. [30] proposed 49 valid features (9 morphological features and 40 textural features) to classify thyroid nodules.

To overcome these concerns about feature extraction and feature selection methods, this article investigated whether the image content can be explained by the *n*-gram model. The *n*-gram model is a classical language model which is based on the probability of the (*n* − 1)-order Markov chain [31]. This model overcomes the language dependence and skips the processing text content by using linguistics [32]. It can extract potential features and take into account the context information of local features; therefore, the *n*-gram model has been widely used in text retrieval and classification, information retrieval [33], probability theory [34], computer language [35], communication theory [36], computational biology [37], etc. Nevertheless, it has not been widely used in the field of medical image classification.

Applying the *n*-gram model to medical image classification is challenging because (1) the text is a one-dimensional vector, whereas the image is a two-dimensional matrix; (2) in the *n*-gram model, the number of all possible word combinations grows exponentially as *n* increases, and these high-dimensional data can lead to dimensional disasters. To solve these problems, we first proposed a method to extract features from grayscale images using the *n*-gram model. This procedure maps the image into a character matrix and then extracts all the *n*-gram character combinations from this matrix sequentially. We then designed a novel feature selection method to reduce the dimensionality of the feature vectors, using the rank sum test and the expected cross-entropy. We validated the feasibility of the proposed approach using two medical datasets, a clinical dataset of ultrasound images of thyroid nodules in China and a human visual optical coherence tomography (OCT) dataset.

The remainder of this paper is structured as follows.  Section 2 gives the definitions and application principles of the basic model.  Section 3 details the proposed method.  Section 4 presents the classification results of two datasets, and Section 5 concludes our work and discusses of the future.

## 2. Method Description

### 2.1. Datasets

In this study, we used two different datasets, hereafter referred to as dataset 1 [38] and dataset 2 [39]. Dataset 1 contained 93 malignant and 415 benign ultrasound images of thyroid nodules, which were provided by the Third Hospital of Hebei Medical University in China. Each image in this dataset represented one patient and contained only one nodule. Dataset 2 was an open-source retinal OCT image dataset, and each image was manually labeled by ophthalmologists. This dataset included volume scans of 45 patients, 15 normal patients, 15 patients with dry AMD, and 15 patients with DME.

### 2.2. *N*-Gram Method

The *n*-gram model is a bag-of-phrases model with *n*-consecutive words as elements. For example, if there is a hexadecimal string “09 EC 84 35 A6 78,” the 2-gram corpus of the string will be “09 EC,” “EC 84,” “84 35,” “35 A6,” and “A6 78.” The feature division process is shown in Figure 1.

In the *n*-gram model [40], the storage space, computation, and computational complexity increase with *n*. Therefore, the default value of *n* is generally 1, 2, and 3. At this point, there are at most *W* + *W*^2^ + *W*^3^ possible word combinations in a text containing *W* words.

### 2.3. Application of *N*-Gram Model in Image Classification

The *n*-gram model is based on three key principles. First, it chooses a part of the dataset as a template. Second, it searches all the segments to get the occurrence frequency of each segment. Finally, it identifies the representative segments of the dataset. To combine the *n*-gram model with image processing tightly and effectively, a new model was proposed in this paper based on the above principles. This model could describe the deeper semantic information of an image with a limited but representative combination of words. The details of the proposed technique are given in the next chapter.

## 3. Method Improvement

### 3.1. Image Preprocessing

The adjacent tissues of thyroid nodules in ultrasound images could interfere with the classification process. The accurate segmentation of the nodule area is conducive to extracting the essential characteristics of pathology. In this paper, the thyroid nodule images were segmented under the guidance of pathologists. On this basis, in order to remove the influence of the nodule shape angle, the longest diameter of the nodule was placed in a horizontal position. The preprocessing procedures are shown in Figure 2.

Speckle noise is the main reason of poor OCT image quality [41]. In this paper, the anisotropic diffusion model is used to denoise retinal OCT images [42, 43]. Another problem is the irregular white edges of the pictures. The solution is to identify the edges and then fill the deselected area with black. The process is shown in Figure 3.

### 3.2. Medical Image Feature Extraction Based on *N*-Gram Model

#### 3.2.1. Transformation from Medical Image to Character Matrix

All images in this paper are represented in grayscale, with values between 0 and 255. This is equivalent to giving a dictionary with 256 words. Then, the number of all possible *n*-grams is 256^*n*^. When “*n* = 1, 2, and 3,” the number is ∑_*n*=1_^3^256^*n*^. Such high-dimensional data can cause information redundancy or noise and dimensional disasters. Therefore, we converted the gray value matrix into a character matrix consisting of 16 letters point by point by using the partition function as shown in the following equation.

(1) $$\begin{array}{c} y_{ij}=\left\{\begin{array}{c} A,x_{ij}\in \left[0,15\right]\\ B,x_{ij}\in \left[16,31\right]\\ \vdots \\ Px_{ij},\in \left[240,255\right] \end{array}\right.,x_{ij}\in X,y_{ij}\in Y. \end{array}$$

In the above formula, *X* is the numerical matrix of the grayscale image, *x*_*ij*_ is the grayscale value at (*i*, *j*)th of *X*, *Y* is the character matrix, and *y*_*ij*_ is the characters located at the  (*i*, *j*)th element of *Y*.

The primary purpose of this step is to convert the image to text to reduce the dimensionality of the image. As shown in equation (3), the corresponding character matrix *Y* can be calculated by equation (1) for a given numerical matrix *X*.

(2) $$\begin{array}{c} X=\left[\begin{array}{ccccccc} 255 & 255 & 255 & \cdots & 255 & 255 & 255\\ \vdots & \vdots & \vdots & \cdots & \vdots & \vdots & \vdots \\ 204 & 174 & 165 & \cdots & 84 & 147 & 223\\ 211 & 196 & 192 & \cdots & 135 & 200 & 249\\ 213 & 200 & 189 & \cdots & 174 & 239 & 255\\ \vdots & \vdots & \vdots & \cdots & \vdots & \vdots & \vdots \\ 255 & 255 & 255 & \cdots & 255 & 255 & 255 \end{array}\right], \end{array}$$

(3) $$\begin{array}{c} \Rightarrow Y=\left[\begin{array}{ccccccc} P & P & P & \cdots & P & P & P\\ \vdots & \vdots & \vdots & \cdots & \vdots & \vdots & \vdots \\ M & K & K & \cdots & F & G & N\\ N & M & M & \cdots & I & M & P\\ N & M & L & \cdots & K & O & P\\ \vdots & \vdots & \vdots & \cdots & \vdots & \vdots & \vdots \\ P & P & P & \cdots & P & P & P \end{array}\right]. \end{array}$$

#### 3.2.2. Feature Extractor Based on *N*-Gram Model

Text retrieval uses a contiguous sequence of *n* words to represent an *n*-gram. Similarly, we collected all *n*-consecutive letters from the character matrix *Y* and defined them as image features. A feature can be interpreted as a combination of grayscale intensities of *n*-consecutive pixels in an image. The detailed process was as follows.

First, a picture in the dataset was converted into a character matrix. Then, all combinations of characters were extracted as a subset of features by letting a window of length *n* characters slide from left to right in each row of the matrix. The above procedure was repeated for each image in the dataset. All the feature subsets were combined to be the set of features of the whole dataset.

The *n*-gram (*n* = 1, 2, and 3) features used to describe the entire dataset in this paper were generated from the training set.

#### 3.2.3. Calculation of Feature Values

The method of calculating the eigenvalues was crucial to the classification ability of the features in the model. So this paper used both Term Frequency (TF) and Term Frequency-Relevance Frequency (TF-RF) [44] methods.

TF represents the frequency of a given word *t*_*i*_ in a document *d*_*j*_. The frequency value was positively correlated with the importance of the word to the text. The word frequency of *t*_*i*_ can be expressed as

(4) $$\begin{array}{c} {tf}_{ij}=\frac{n_{ij}}{\sum_{k}n_{kj}}. \end{array}$$

In the above formula, *n*_*ij*_ is the number of occurrences of word *t*_*i*_ in document *d*_*j*_ and ∑_*k*_*n*_*kj*_ is the sum of the number of occurrences of all words in document *d*_*j*_.

The basic idea of RF is that the higher the concentration of a high-frequency term in the positive category, the greater its contribution to selecting positive samples from the negative category. For the word *t*_*i*_ in the corpus, its formula is expressed as

(5) $$\begin{array}{c} {rf}_{i}=\log_{2}\left(2+\frac{a}{\max\left(1,c\right)}\right). \end{array}$$

In the above formula, *a* is the number of documents containing the word *t*_*i*_ and belonging to the positive category and *c* is the number of documents containing the word *t*_*i*_ and belonging to the negative category. Considering the imbalance of medical image samples, the final TF-RF calculation formula is as follows:

(6) $$\begin{array}{c} tf\_{rf}_{i}={tf}_{i}*\log_{2}\left(2+\frac{N}{P}*\frac{a}{\max\left(1,c\right)}\right). \end{array}$$

In the above formula, *P* is the total number of positive categories in the training set and *N* is the total number of negative categories in the training set.

### 3.3. Feature Selection

A new feature selection method with two steps was applied to remove redundant and irrelevant features. The detailed steps were as follows. In step one, a rank sum test [45] was performed for each feature using the training set data, and only the features with significant differences were retained, with the following assumptions.

(7) $$\begin{array}{c} \begin{array}{c} \text{H}0:\text{The two populations have equal variance or spread},\\ \text{H}1:\text{The two populations are independent of one another}, \end{array}\alpha =0.05. \end{array}$$

If the calculated *p* value for a feature was less than *α*, H0 was rejected, meaning that the difference between the features on positive and negative samples was statistically significant. Only such features were chosen for subsequent analysis.

In step two, based on the previous step, the importance of each feature was measured using the expected cross-entropy (ECE) [46], and the features were sorted in descending order by entropy value. The formula was shown as follows.

(8) $$\begin{array}{c} \text{ECE}=p\left(t_{i}\right)*\underset{j}{\sum }p\left(\left.C_{j}\right|t_{i}\right)*\log_{2}\left(\frac{p\left(\left.C_{j}\right|t_{i}\right)}{p\left(C_{j}\right)}\right), \end{array}$$

where *C*_*j*_ is the *j*th category, *p*(*t*_*i*_) is the sample frequency of feature *t*_*i*_, and *p*(*C*_*j*_|*t*_*i*_) is the sample frequency of category *C*_*j*_ under the condition of feature *t*_*i*_.

### 3.4. Classification

On each dataset, we trained two different classifiers, the Support Vector Machine (SVM) [47, 48] and Back Propagation (BP) neural network [49], and ran the classification experiments using 10-fold cross-validation. All experiments were performed using MATLAB R2019a.

The first experiment is to diagnose whether a nodule is benign or malignant based on dataset 1. We used the receiver operating characteristic (ROC) curve as well as the area under the ROC curve (AUC) to evaluate the performance of the method in this experiment. The closer the ROC curve is to the upper left corner, the closer the AUC value is to 1, indicating better performance [50]. The second experiment is to diagnose whether the type of fundus lesion is AMD, DME, or normal based on dataset 2. Its classifier is a ternary-classifier consisting of three small two-classifiers. The classification result is determined by the vote of each subclassifier. The parameter settings of all classifiers are shown in Table 1, and other parameters not listed in the table were default values.

## 4. Discussion

According to the characteristics of medical images, an improved classification algorithm based on the *n*-gram model was proposed in this paper. The algorithm has been described in detail previously. The core steps of the algorithm were described here in conjunction with specific experiments, as shown in Algorithm 1.

Take the experiment with dataset 1 as an example. First, the basic feature set *T* and the feature matrix *T*_*x*_ are obtained from the training set as described in Section 3.2. Second, a subset *T*′ of *T* and a submatrix *T*_*x*_′ of *T*_*x*_ are selected, according to the method in Section 3.4. Next, we train the classifier using *T*_*x*_′. Finally, we predict the labels of the test set samples, as shown in Step 3 in Algorithm 1.

### 4.1. Experimental Results of Dataset 1

The impact of two eigenvalue calculation methods and four feature dimensions on classification was explored using dataset 1. The specific work is as follows. First, the eigenvalues of the training set were calculated using the two equations TF and TF-RF introduced in Section 3.2.3 to obtain two feature matrices. Second, the same two-step operation to select the submatrices to control the dimensionality was performed for these two matrices as follows. The first step was to calculate the ECE values of the features after selecting the features with the rank sum test according to Section 3.3 The second step was that features were ranked according to ECE values, and 100%, 75%, 50%, and 25% features were selected from the highest to the lowest. After the above work, eight feature submatrices were obtained as the input matrix for training the classifier.

Based on the average of the 10-fold cross-validation results, we observed that the number of valid features was less than the number of all features, and the method of calculating the feature values had an impact on the validity of the features. The variation of feature dimensions is shown in Table 2.

In summary, we conducted a total of 160 experiments on dataset 1, and the cross-validation results are shown in Figure 4. The best diagnostic result was achieved in the experiment with an AUC of 0.989 under the condition that the input was all valid features, the classifier was an SVM, and TF was used to calculate the eigenvalues.

Overall, this experiment showed that SVM outperformed the BP neural network for classification and TF outperformed TF-RF for discriminating samples. It also showed that when 25% of the valid features were selected, the AUC fluctuated only 0.5% from the optimal level, which could balance feature dimensionality and accuracy. The average compression rate of the algorithm for this dataset is 4.7% based on the 126M original size of the dataset and the 5.91M average size of the feature matrix in the 10-fold cross-validation. The average computation time for this experiment is 267 ms per image.

### 4.2. Experimental Results of Dataset 2

The triple classification experiment for dataset 2 selected 25% of the valid features as input to the SVM and BP neural network classifiers, and its 10-fold cross-validation results are shown in Table 3. When the formula for calculating feature values was TF-RF and the classifier was SVM, this experiment achieved the best diagnostic result of correctly identifying 86.667% of AMD patients, 93.333% of DME patients, and 93.333% of normal patients.

Overall, this experiment shows that SVM outperforms the BP neural network for classification and TF-RF discriminates the samples better than TF. The average compression rate of the algorithm for this dataset was calculated to be 6.7% based on the original size of the dataset of 946M and the average size of the feature matrix of 10-fold cross-validation of 63M. The average computation time for this experiment is 760 ms per image.

## 5. Conclusions and Future Works

In this paper, a new medical image classification method is proposed and experimentally validated using two datasets. Dataset 1 is clinically unbalanced ultrasound images of thyroid nodules, and dataset 2 is OCT images of the fundus. The algorithm showed good classification performance on both datasets, which reflected its generalization ability.

The algorithm performs the rank sum test for each feature to ensure its robustness. Therefore, the performance of the algorithm remains stable under the condition that the preprocessing is coarse, and only denoising is performed without steps such as histogram equalization, brightness correction, and geometric transformation. One of the key works is to propose an algorithm for extracting image features based on the *n*-gram model, which maps the image into a character matrix and then applies a text-processing approach to extract image features instead of relying on traditional morphological and texture features. Another key work is to reduce the number of features by selecting features in two steps. The intent of these two works is to express the deep semantic information of the image with the appropriate number of features. In conclusion, the method is simple and efficient compared to more complex models and has important theoretical implications and potential for clinical applications.

In the future, we will try to optimize the model in several aspects such as spatial information [51, 52], distribution of features [53, 54], clustering of features [55, 56], selection of features [57], and evaluation of features [58]. We explore the use of some representative computational intelligence algorithms [59, 60] to solve the problem, such as monarch butterfly optimization (MBO), earthworm optimization algorithm (EWA), elephant herding optimization (EHO), moth search (MS) algorithm, slime mould algorithm (SMA), hunger games search (HGS), Runge-Kutta optimizer (RUN), colony predation algorithm (CPA), and Harris hawks optimization (HHO).

## Figures and Tables

**Figure 1:** Hex string 2-gram partition example.

**Figure 2:** Ultrasonic image preprocessing of thyroid nodules. (a) The original image. (b) Image after removing adjacent tissues of nodules. (c) Image after adjusting nodule angle.

**Figure 3:** Retinal OCT image preprocessing. (a) The original image. (b) The preprocessed image.

**Figure 4:** The results of 10-fold cross-validation. (a) The classifier with SVM and TF achieves the best AUC of 0.989 using all features as inputs. (b) The classifier with BP and TF achieves the best AUC of 0.981 using 25% features as inputs. (c) The classifier with SVM and TF-RF achieves the best AUC of 0.978 using all features as inputs. (d) The classifier with BP and TF-RF achieves the best AUC of 0.977 using 25% features as inputs.

**Algorithm 1:** Proposed algorithm.

**Table 1:** Parameter settings for both classifiers.

libsvm		newff			
c	g	Si	Epochs	Goal	lr
10	0.01	3, 6, 3	100	1*e*-5	0.01

**Table 2:** Characteristic dimension.

Mode	Essential feature	Distinguishing feature			
		100%	75%	50%	25%
TF	3590	1463	1098	732	366
TF-RF	3590	1338	1004	669	335

**Table 3:** Fraction of correctly classified during cross-validation.

Class	TF-SVM	TF-BP	TF-RF-SVM	TF-RF-BP
AMD	13/15 = 86.667%	13/15 = 86.667%	13/15 = 86.667%	12/15 = 80.000%
DME	13/15 = 86.667%	11/15 = 73.333%	14/15 = 93.333%	12/15 = 80.000%
Normal	14/15 = 93.333%	14/15 = 93.333%	14/15 = 93.333%	14/15 = 93.333%

## Data Availability

We have uploaded the source code to the GitHub (https://github.com/Wanggf618/Medical-Image-Classification-Algorithm-Based-on-N-Gram-Model.git).
